The article "A Novel Hybrid Algorithm for Multiobjective Location-Allocation Problem in Emergency Logistics" was retracted in 2023. Reasons: unreliable results or conclusions; concerns about the data; concerns about the results or conclusions; concerns about the peer review.

# A Novel Hybrid Algorithm for Multiobjective Location-Allocation Problem in Emergency Logistics

**DOI:** 10.1155/2021/1951161

**Published:** 2021-11-28

**Authors:** Hongrui Chu, Yahong Chen

**Affiliations:** ^1^School of Management and Engineering, Capital University of Economics and Business, Beijing 100070, China; ^2^Beijing Intelligent Logistics System Collaborative Innovation Center, School of Information, Beijing Wuzi University, Beijing 101149, China

## Abstract

Increased frequency of disasters keeps reminding us of the importance of effective resource distribution in postdisaster. To reduce the suffering of victims, this paper focuses on how to establish an effective emergency logistics system. We first propose a multiobjective optimization model in which the location and allocation decisions are made for a three-level logistics network. Three objectives, deprivation costs, unsatisfied demand costs, and logistics cost, are adopted in the proposed optimization model. Several cardinality and flow balance constraints are considered simultaneously. Then, we design a novel effective IFA-GA algorithm by combining the firefly algorithm and genetic algorithm to solve this complex model effectively. Furthermore, three schemes are proposed to improve the effectiveness of the IFA-GA algorithm. Finally, the numerical results provide several insights on the theory and practice of relief distribution, which also illustrate the validity of the proposed solution algorithm.

## 1. Introduction

Large-scale natural or man-made disasters, such as the 2010 Haitian Earthquake, the 2011 tsunami in Japan, the civil war in Syria, and the 2019 coronavirus disease, have occurred frequently throughout the world, resulting in tremendous consequences of enormous casualties and property losses. The world has witnessed a steadily increased number in both disasters and affected people since the 1900s. After large-scale disasters, a great need for medical and daily supplies will be invoked in the affected areas, which lack adequate relief resources. Thus, the rapid distribution of external commodities is critical to mitigating the losses caused by disasters. Therefore, emergency logistics has received wide attention from both practical managers and scholars [1]. However, how to design an efficient emergency logistics system is a big challenge [2]. Before the last decade, most research on emergency management focused on the responses of public servants, government agencies, and insurance firms in times of crisis [3]. Emergency logistics, also commonly known as humanitarian logistics, is emerging and becoming a hot spot of operations management in the recent decade.

In most of the current related research, emergency logistics problems are studied based on the analytical formulations of the traditional commercial sector, unlike the commercial scenario, whose decision objective is to minimize the logistics cost. In emergency relief cases, the scientific community is encouraged to provide effective logistics systems to reduce human suffering. Therefore, the adapted objectives in commercial and emergency logistics are radically different. The modified analytical formulations of the traditional logistics are not very suitable for emergency logistics problems [4].

The article "A Novel Hybrid Algorithm for Multiobjective Location-Allocation Problem in Emergency Logistics" was retracted in 2023. Reasons: unreliable results or conclusions; concerns about the data; concerns about the results or conclusions; concerns about the peer review.

To derive an appropriate objective function for emergency logistics, Holguín-Veras et al. [5] incorporated welfare economic principles into emergency management and introduced the deprivation costs, which express the economic value of human suffering caused by a lack of access to resources or services. Since then, some studies using deprivation costs have been conducted in the emergency logistics field [6]. For example, Pérez-Rodríguez and Holguín-Veras [7] developed an inventory-allocation-routing model for the optimal critical supplies by minimizing logistics and social costs. Ismail [3] studied a relief distribution problem by considering the logistics and deprivation costs. Some other papers also considered human suffering in the emergency logistics field. Chapman and Mitchell [8] studied the distribution centers selection problem by minimizing the suffering of the population. Cotes and Cantillo [9] developed a facility location model for prepositioning supplies in preparation for disasters. Their formulation considers deprivation costs in the objective function. Rivera-Royero et al. [10] proposed a dynamic model to serve rescue demand. They considered the level of urgency of demand points. Moreno et al. [11] presented a novel model to optimize location, transportation, and fleet sizing for emergency logistics with considering deprivation costs. Cantillo et al. [12] assessed transportation network vulnerability from logistical costs and deprivation costs. Zhu et al. [13] studied the emergency relief routing optimization problem considering injured degree and deprivation cost.

Similar to the above literature, we adopt the deprivation costs to characterize human suffering in this paper. We study a location-allocation problem of emergency logistics. Three objectives, deprivation costs, unsatisfied demand losses, and logistics costs, are adopted in the proposed optimization model. The fairness objective of this paper equalizes the supplies between affected areas, which has the same purpose as unmet demand minimization in [14]. In addition, our literature also lies in the stream of multiobjective programming, which is widely used to solve emergency optimization problems. Sun et al. [15] proposed a robust optimization model to decide the facility location, resource allocation, and casualty transportation in a three-level rescue chain composed of casualty clusters, temporary facilities, and general hospitals. Their objectives are to minimize the total Injury Severity Score (ISS) and logistics cost. Zhou et al. [2] studied the multiperiod dynamic emergency resource scheduling problem by a proposed multiobjective optimization model. Cao et al. [16] proposed a multiobjective nonlinear programming model for resource distribution regarding the beneficiary perspective on sustainability. The model is solved by maximizing the lowest victims' perceived satisfaction and minimizing the largest deviation of victims' perceived satisfaction. Çelik et al. [17] studied the stochastic debris clearance problem among postdisaster operations. They determined a sequence of roads to clear with the goal of maximizing satisfied relief demand. Gralla et al. [18] developed a method to value the objective functions of emergency logistics based on expert preferences over five key attributes. They found that the amount of cargo delivered is the most valued objective and cost the least important. In a similar vein, we conduct the optimization problem based on a three-level emergency logistics network. Considering the complexity of reality, we formulate the problem by a multiobjective mixed-integer nonlinear programming with cardinality and flow balance constraints.

The article "A Novel Hybrid Algorithm for Multiobjective Location-Allocation Problem in Emergency Logistics" was retracted in 2023. Reasons: unreliable results or conclusions; concerns about the data; concerns about the results or conclusions; concerns about the peer review.

Most optimization problems of emergency logistics are hard to solve effectively by exact algorithms, especially in the limited available time. In such situations, adopting a metaheuristic algorithm is imperative [19]. The third related literature stream of this paper is algorithm design. Zhou et al. [2] designed an evolutionary algorithm based on decomposition (MOEA) to solve a multiobjective multiperiod dynamic emergency resource scheduling problem. Cao et al. [16] adopted genetic algorithm to solve a relief distribution model. Haghi et al. [20] proposed a multiobjective location and transportation programming model, which is solved by a nondominant sorting genetic algorithm. Eisenhandler and Tzur [21] modeled a food rescue problem as a routing resource allocation problem with the equitable allocations objective. They presented a heuristic approach based on the large neighborhood search framework to solve the model. Zhang et al. [22] determined the truck and drone routes in a humanitarian relief network by combining column generation and tabu search algorithms. This paper designs a metaheuristic algorithm named IFA-GA by combining the firefly algorithm and genetic algorithm. Some improved schemes are embedded into IFA-GA to obtain better solutions.

The article "A Novel Hybrid Algorithm for Multiobjective Location-Allocation Problem in Emergency Logistics" was retracted in 2023. Reasons: unreliable results or conclusions; concerns about the data; concerns about the results or conclusions; concerns about the peer review.

The contributions of this paper can be summarized as follows: first, we propose a new multiobjective location-allocation optimization model for emergency logistics, in which deprivation costs, fairness, and operation costs are considered. The numerical results show that deprivation costs have a significant effect on location decisions. Second, we design a new IFA-GA algorithm based on the combination of the firefly algorithm and genetic algorithm. Three schemes, population initialization, search strategy, and update mechanism of population, are proposed to improve IFA-GA. The computational results illustrate that the proposed IFA-GA has better solving performance than the other algorithms.

The remainder of this paper is organized as follows: Section 2 presents some presumptions and notations. The detailed descriptions of the three objective functions and model formulation are also given in Section 2.  Section 3 develops the hybrid IFA-GA algorithm for solving the proposed model and gives the improved schemes.  Section 4 conducts numerical studies and analyses. Finally, Section 5 presents conclusions and future work.

## 2. Problem Description and Formulation

In this section, we first give some presumptions and notations. Then, three relief-related objective functions are proposed to represent human suffering, fairness, and logistics cost. Finally, we present a multiobjective location and resource allocation model for three-level emergency logistics.

### 2.1. Presumptions and Notations

Emergency supplies mainly come from two sources: local rescue warehouses or external dispatching. Local rescue warehouses can provide supplies immediately after disasters occur, but the amount is limited. External dispatching mainly comes from the Strategic National Stockpile (SNS), which integrates different parties' resources and provides the primary resources to the affected areas by railway or airplane in the subsequent relief phase. In this paper, we consider an emergency logistics problem in the second case. Most emergency logistics systems have a three-tier structure, including SNS, regional transfer center (RTC), and local distribution point (LDP). In reality rescue practice, large amounts of emergency resources must be transported from SNS to affected points as soon as possible. To improve the efficiency of the rescue, RTCs are proposed as hubs to bridge SNS and LDP. This work proposes a joint facility location and resource allocation model for this three-level emergency logistics system. Some assumptions used in our model are as follows:

1. There are one SNS, some RTCs, and a fixed number of LDPs. The resources are first transported from SNS to RTCs and then transported from RTCs to LDPs. LDPs are equivalent to affected points that have resource demands. SNS, RTCs, and LDPs have enough capacity to store resources. The capacity constraints are ignored in our optimization model.
2. The demand quantity of resources in each affected point can be predicted, and the total available quantity of resources is also known.
3. The rescue resources are transported by trucks. Moreover, there are enough available trucks in each supply point.
4. The locations of RTCs are decided in the postdisaster phase. After establishing RTCs, all roads from RTCs to SNS and LDPs are fixed. This work does not consider the uncertainty of road networks. Therefore, the delivery time between two supply points is determined by the speed of the truck.
5. The rescue demand has an additional time-related attribute. If the actual delivery time exceeds the required threshold, the deprivation costs of victims will be invoked to represent the economic valuation of the human suffering associated with a lack of access to a good or service.

The article "A Novel Hybrid Algorithm for Multiobjective Location-Allocation Problem in Emergency Logistics" was retracted in 2023. Reasons: unreliable results or conclusions; concerns about the data; concerns about the results or conclusions; concerns about the peer review.

The RTCs are established in selected reasonable sites the first time after the disaster occurs. In commercial logistics, RTCs can quickly move goods from the central warehouse, manufacturers to retailers. In emergency logistics, large-scale disaster is characterized by a wide range of affected points, great demand, and long duration. Therefore, the appropriate location of RTCs has a more critical role in improving the transport efficiency of resources. With the above assumptions, the location decision of RTCs, the allocation decisions from SNS to RTCs and from RTCs to LDPs will be studied in our proposed multiobjective optimization model. The notations used in the following text are listed as follows:

- *O*: the SNS point;
- *I*: the candidate location set of RTCs, *i*=1,2,…, *I*;
- *J*: the location set of LDPs, *j*=1,2,…, *J*;
- *d*_*Oi*_: the distance from SNS *O* to RTC candidate *i*;
- *d*_*ij*_: the distance from RTC candidate *i* to LDP *j*;
- *C*_*OI*_: the unit transport cost from SNS to RTC;
- *C*_*IJ*_: the unit transport cost from RTC to LDP;
- *C*_*i*_: the construction cost of RTC *i*;
- *CV*_*i*_: the unit operation cost of RTC *i*, *CV*_*i*_ multiplied by inventory equal to the total operation cost of RTC *i*;
- *D*_*j*_: the demand quantity of LDP *j*;
- *Q*_*o*_: the initially available quantity of the resource in SNS;
- *Q*_*i*_: the initially available quantity of the resource in RTC *i*;
- *π*_*jt*_: the unit deprivation cost of each victim in LDP *j* at time *t*;
- *δ*_*j*_: the deprivation costs of LDP *j* at time *t*;
- *lo*_*j*_: the loss function of unsatisfied demand of LDP *j*;
- OC: the total operation cost of emergency logistics;
- *t*_*ij*1_: the first delivery time of resources from RTC *i* to LDP *j*;
- *t*_*ij*2_: the second delivery time of resources from RTC *i* to LDP *j*;
- *v*: the speed of truck;
- *z*_*i*_: 0–1 variables, if candidate *i* is selected as RTC, *z*_*i*_=1, else, *z*_*i*_=0;
- *x*_*oi*_: the allocated quantity of emergency resources from SNS to RTC *i*;
- *y*_*ij*1_: the first allocated quantity of emergency resources from RTC *i* to LDP *j*;
- *y*_*ij*2_: the second allocated quantity of emergency resources from RTC *i* to LDP *j*;
- *ɛ*_*ij*_: auxiliary variable, *ɛ*_*ij*_=1 if RTC *i* provides resources to LDP *j*, else *ɛ*_*ij*_=0.

The article "A Novel Hybrid Algorithm for Multiobjective Location-Allocation Problem in Emergency Logistics" was retracted in 2023. Reasons: unreliable results or conclusions; concerns about the data; concerns about the results or conclusions; concerns about the peer review.

### 2.2. Multiobjective Optimization Model

There are three objectives in our model that reflect three service levels of emergency logistics: (1) minimizing the total deprivation costs of victims, (2) minimizing the loss of unsatisfied demand, and (3 minimizing the total cost of the emergency logistics system. The formulations consider a relief group that first delivers critical supplies from SNS to RTCs and then delivers goods from RTCs to demand nodes. Furthermore, RTCs also have a limited initial inventory of critical supplies. Therefore, there are twice transportations from RTC *i* to LDP *j* if RTC *i* is selected as a hub to supply LDP *j*. RTC *i* first provides resources by its own inventory. The first resources reach LDP *j* at time *t*_*ij*1_. Then, RTC *i* transfers the second resources which come from SNS and arrive at LDP *j* at time *t*_*ij*2_. During a planning horizon *T*, the relief group's decisions are which RTCs should be selected, how much, and when to deliver to the demand nodes in need of supplies.

#### 2.2.1. The Deprivation Costs

Human suffering is one of the critical factors in humanitarian logistics. The theory of deprivation costs [5] provides an excellent method to bring human suffering factors into the decision objective. Conceptually, deprivation cost is the economic value of human suffering caused by a lack of access to resources or services. Suppose LDPs at which identical individuals experience the same unit deprivation cost *π*(*t*) at time *t*. According to the theory of deprivation costs, the deprivation costs function *δ*_*j*_ is discontinuous, increases with deprivation time, and then drops to zero when a delivery large enough to fulfill the needs of all individuals is received. The total deprivation costs at node *j* are equal to the aggregation of individual costs:

(1) $$\begin{array}{c} \delta_{j}=\pi \left(t_{ij1}\right)\min\left(D_{j},y_{ij1}\right)+\pi \left(t_{ij2}\right)\min\left(\max\left(D_{j}-y_{ij1},0\right),y_{ij2}\right)+\pi \left(T\right)\max\left(D_{j}-y_{ij1}-y_{ij2},0\right), \end{array}$$

where *t*_*ij*1_ is dependent on the distance between RTC *i* and LDP *j*. *t*_*ij*2_ is dependent on the distance from SNS to LDP *j* via RTC *i*. The first part of *δ*_*j*_ is the deprivation costs of the satisfied demand in the first supply. The second part of *δ*_*j*_ is the deprivation costs of the satisfied demand in the second supply. The third part of *δ*_*j*_ is the deprivation costs of the remaining unsatisfied demand at the end.

The article "A Novel Hybrid Algorithm for Multiobjective Location-Allocation Problem in Emergency Logistics" was retracted in 2023. Reasons: unreliable results or conclusions; concerns about the data; concerns about the results or conclusions; concerns about the peer review.

It should be noted that the beneficiaries had already experienced a deprivation cost at time *t* < *t*_*ij*1_. Therefore, the classical deprivation costs theory evaluates the cumulative cost function up to time *T*. For simplification, this work only considers the deprivation costs at the arrival times of supplies and the end time of the period. The unite deprivation cost *π*(*t*) is increasing convex function with respect to *t*, 0 < *t* ≤ *T*. In this paper, we use a quadratic function *π*(*t*)=*at*^2^ to specify deprivation cost and *a* is a cost coefficient. Thus, we can easily obtain the total deprivation costs at the end of period *T*, which can be expressed as

(2) $$\begin{array}{c} \sum_{j\in J}\delta_{j}=\sum_{i\in I,j\in J}at_{ij1}^{2}\min\left(D_{j},y_{ij1}\right)+at_{ij2}^{2}\min\left(\max\left(D_{j}-y_{ij1},0\right),y_{ij2}\right)+aT^{2}\max\left(D_{j}-y_{ij1}-y_{ij2},0\right). \end{array}$$

#### 2.2.2. The Loss of Unsatisfied Demand

In the context of emergency rescue, decision-makers should try their best to meet the supplies needs in each affected point, but the goods are inadequate at the first time. Therefore, another important objective in emergency logistics is to keep fairness. In this work, we provide a loss function of unsatisfied demand to evaluate the fairness of rescue. The loss function *lo*_*j*_ is an *S* type curve of unsatisfied demand in LDP *j*. This reflects that the unsatisfied demand has a learning effect on the emergency service level. If the unsatisfied demand takes the maximum value, the loss function becomes constant, and no more losses will occur. In addition, developed regions tend to be densely populated, which have more severe consequences if emergency demands are not met. Thus, the demand quantity is considered in the loss function, which can be given by

(3) $$\begin{array}{c} lo_{j}=\max\left(D_{j}-y_{ij1}-y_{ij2},0\right)P\left(h_{j}\right), \end{array}$$

where *P*(*h*_*j*_)=*be*^(−*h*_*j*_/(1 − *h*_*j*_))^ and *h*_*j*_=(∑_*i*∈*I*_*y*_*ij*1_+*y*_*ij*2_/*D*_*j*_). *h*_*j*_ is the proportion of satisfied demand in LDP *j*. Obviously, 1 − *h*_*j*_ is the ratio of unsatisfied demand. *P*(*h*_*j*_) is related to service level, which converges to loss upper bound *b* if *h*_*j*_ tends to 0, and 0 if *h*_*j*_ tends to 1. Thus, we use the above loss function to quantify the fairness in this paper. The total unsatisfied demand loss of emergency logistics is given as follows:

(4) $$\begin{array}{c} \underset{j\in J}{\sum }lo_{j}=\underset{i\in I,j\in J}{\sum }\max\left(D_{j}-y_{ij1}-y_{ij2},0\right)P\left(h_{j}\right). \end{array}$$

The article "A Novel Hybrid Algorithm for Multiobjective Location-Allocation Problem in Emergency Logistics" was retracted in 2023. Reasons: unreliable results or conclusions; concerns about the data; concerns about the results or conclusions; concerns about the peer review.

#### 2.2.3. The Operation Cost

The operation cost of emergency logistics includes three parts: the construction cost of RTCs, the transport cost, and the inventory holding cost in RTCs. In the setting of this paper, the SNS already exists before disasters occur. The LDPs will distribute the relief resources as soon as they are received. Thus, we only consider the holding cost of RTCs because they are newly built. Then, the operation cost objective can be given by

(5) $$\begin{array}{c} \text{OC}=\sum_{i\in I}\left[z_{i}C_{i}+C_{Oi}d_{oi}x_{oi}+\sum_{j\in J}C_{ij}d_{ij}\left(y_{ij1}+y_{ij2}\right)+CV_{i}\left(x_{oi}+Q_{i}\right)\right]. \end{array}$$

### 2.3. Mathematical Formulation

Based on the above analysis, we suppose that the emergency manager's goals are to minimize the deprivation costs, the loss of unsatisfied demand, and the operation cost. Without loss of generality, we adopt two weight parameters *α* and *β*(0 < *α*, *β*, 1 − *α* − *β* < 1) to simplify this multiobjective optimization to scalar objective optimization. Meanwhile, the manager also needs to consider some realistic constraints, such as path constraint and capacity constraints. Then, the logistics optimization model is formulated as follows:

(6) $$\begin{array}{c} \min\alpha \sum_{j\in J}\delta_{j}+\beta \sum_{j\in J}lo_{j}+\left(1-\alpha -\beta \right)\text{OC}, \end{array}$$

(7) $$\begin{array}{c} \text{s.t. }\delta_{j}=\sum_{i\in I}at_{ij1}^{2}\min\left(D_{j},y_{ij1}\right)+at_{ij2}^{2}\min\left(\max\left(D_{j}-y_{ij1},0\right),y_{ij2}\right)+aT^{2}\max\left(D_{j}-y_{ij1}-y_{ij2},0\right),\;\forall j\in J, \end{array}$$

(8) $$\begin{array}{c} lo_{j}=\max\left(D_{j}-y_{ij1}-y_{ij2},0\right)P\left(h_{j}\right),\;\forall j\in J, \end{array}$$

(9) $$\begin{array}{c} P\left(h_{j}\right)=be^{\left(-h_{j}/1-h_{j}\right)},\;\forall j\in J, \end{array}$$

(10) $$\begin{array}{c} h_{j}=\frac{\sum_{i\in I}y_{ij1}+y_{ij2}}{D_{j}},\;\forall j\in J, \end{array}$$

(11) $$\begin{array}{c} \text{OC}=\sum_{i\in I}\left[z_{i}C_{i}+C_{Oi}d_{oi}x_{oi}+\sum_{j\in J}C_{ij}d_{ij}\left(y_{ij1}+y_{ij2}\right)+CV_{i}\left(x_{oi}+Q_{i}\right)\right], \end{array}$$

(12) $$\begin{array}{c} t_{ij1}=\frac{d_{ij}}{v},\;\forall i\in I,j\in J, \end{array}$$

(13) $$\begin{array}{c} t_{ij2}=\frac{d_{ij}+d_{oi}}{v},\;\forall i\in I,j\in J, \end{array}$$

(14) $$\begin{array}{c} \sum_{i\in I}\in_{ij}=1,\;\forall j\in J, \end{array}$$

(15) $$\begin{array}{c} \sum_{j\in J}\in_{ij}y_{ij1}=Q_{i},\;\forall i\in I, \end{array}$$

(16) $$\begin{array}{c} \sum_{j\in J}\in_{ij}y_{ij2}=x_{oi},\;\forall i\in I, \end{array}$$

(17) $$\begin{array}{c} y_{ij1}\leq M\in_{ij}z_{i},\;\forall i\in I,j\in J, \end{array}$$

(18) $$\begin{array}{c} y_{ij2}\leq M\epsilon_{ij}z_{i},\;\;\forall i\in I,j\in J, \end{array}$$

(19) $$\begin{array}{c} \epsilon_{ij}\leq z_{i},\;\forall i\in I,j\in J, \end{array}$$

(20) $$\begin{array}{c} \sum_{i\in I,j\in J}\in_{ij}\left(y_{ij1}+y_{ij2}\right)=\min\left(Q_{o}+\sum_{i\in I}Q_{i},\sum_{j\in J}D_{j}\right), \end{array}$$

(21) $$\begin{array}{c} x_{oi}\leq Mz_{i},\;\forall i\in I, \end{array}$$

(22) $$\begin{array}{c} \sum_{i\in I}x_{oi}=Q_{o}, \end{array}$$

(23) $$\begin{array}{c} z_{i},{ɛ}_{ij}\in \left\{0,1\right\},\;\forall i\in I,j\in J, \end{array}$$

(24) $$\begin{array}{c} x_{oi},y_{ij1},y_{ij2}\in R^{+},\;\forall i\in I,j\in J. \end{array}$$

The objective function shown in equation (6) has been described detailedly in the above. Constraints (7), (8), and (11) show the computational formulas of the three objectives, respectively. Constraints (9) and (10) describe the loss function and the satisfied demand rate used to calculate the second objective. Constraints (11) and (12) describe the relationship between transport distance and delivery time. Constraint (14) restricts that each LDP can only receive goods from one RTC. Constraints (15) and (16) balance the flows of resources in each RTC for the first and second deliveries. Constraints (17) and (18) guarantee that RTC *i* can provide relief supplies to LDP *j* only if *i* has been selected and *j* is allocated to it. Here, *M* is a sufficiently large number. Constraint (19) ensures that only a selected RTC can provide emergency supplies to LDPs. Constraint (20) indicates that all goods need to be shipped if the supply is less than demand; else, the delivered quantity is equal to demand. Constraint (21) ensures that only the selected RTC can receive goods from SNS. Constraint (22) indicates the flow balance of resources in SNS. Finally, constraints (23) and (24) define the decision variables.

The article "A Novel Hybrid Algorithm for Multiobjective Location-Allocation Problem in Emergency Logistics" was retracted in 2023. Reasons: unreliable results or conclusions; concerns about the data; concerns about the results or conclusions; concerns about the peer review.

## 3. A Hybrid Heuristic Solution Approach

The proposed model is one of the location-allocation type problems, most of which is NP-hard. Therefore, the optimal solution of the proposed model is difficult to be obtained in a short time. However, the actual emergency decision-making often has higher requirements on timeliness, which inspires us to adopt metaheuristic algorithms. This section combines an improved firefly algorithm with a genetic algorithm to design a new hybrid algorithm called IFA-GA. Furthermore, some schemes are also proposed to increase the solution quality.

### 3.1. The Firefly Algorithm (FA)

FA is a nature-inspired swarm-based optimization algorithm proposed by Yang [23], which is designed to imitate the natural phenomenon of fireflies. FA supposes that all fireflies are homogeneous. Each firefly will be attracted and move close to a brighter firefly. If there are no brighter fireflies nearby, the firefly will move randomly. For an optimization problem, fireflies represent feasible solutions. The brightness of the firefly has a positive relationship with its objective value.

Similar to some other metaheuristic algorithms, FA also successfully implements the exploration and exploitation steps to solve optimization problems. The exploration step is carried out by the movement of fireflies from the current position to a brighter position. The exploitation step is realized by the random movements of the rest fireflies. Suppose *X*_*n*_ is a solution (firefly) in the *n*-th iteration of FA, the update movement equation of this firefly is

(25) $$\begin{array}{c} X_{n+1}=X_{n}+\beta_{0}e^{-\gamma r^{2}}\left({\tilde{X}}_{n}-X_{n}\right)+\alpha_{n}\varepsilon_{n}, \end{array}$$

where *β*_0_ is the maximum attractiveness between fireflies. *r* is the Euclidean distance between two fireflies ${\tilde{X}}_{n}$ and *X*_*n*_. *γ* is the light absorption coefficient that adjusts the change of attraction. *α*_*n*_ is a weight coefficient between [0,1], and *ε*_*n*_ is a random vector in [0,1].

### 3.2. The Genetic Algorithm (GA)

GA is initially motivated by the Darwinian principle of evolution through natural selection and genetic mechanisms, which has been successfully applied to a wide range of real-world problems of significant complexity. Unlike the iterative update mechanism in other algorithms, GA derives a new solution by operating the existing solutions directly. There are two genetic operators in GA: crossover and mutation. A typical design for a classical GA can be given as follows:

1. Initialize a population in which chromosomes are generated randomly.
2. Calculate the fitness of each chromosome in the population.
3. Generate new chromosomes by the following steps: (a) select two chromosomes using the proportional fitness selection, and then cross the selected chromosomes to obtain a child chromosome; (b) select one chromosome using the proportional fitness selection, and apply uniform mutation to it with a mutation rate to produce another child chromosome.
4. Update the population. Add new chromosomes to the population and dispose of the worst chromosomes to maintain the size of the population.
5. If the stopping criteria have not been met, return to Step 2.

The article "A Novel Hybrid Algorithm for Multiobjective Location-Allocation Problem in Emergency Logistics" was retracted in 2023. Reasons: unreliable results or conclusions; concerns about the data; concerns about the results or conclusions; concerns about the peer review.

GA is first proposed by Holland [24] to solve computationally intractable problems. The development and success of GAs have greatly enriched the computational approaches for the optimization problem. Particularly, GA is very suitable for combinatorial optimization problems whose structure and character can avoid the tedious coding and decoding works of chromosomes.

### 3.3. The IFA-GA Algorithm

FA has a good convergence speed due to the attraction of fireflies. However, the solution of FA may fall into a local optimum because of its limited exploration capability, especially when the fireflies encounter extreme values. In contrast, GA can explore the solution space widely due to the crossover and mutation operators. However, the convergence rate of GA is relatively slow due to the lack of directionality. Fortunately, both FA and GA have specific and understandable procedures which are easy to implement. Furthermore, both of them are suitable to be hybridized with other optimizers due to their multimodalities. Inspired by these privileges, we introduce an IFA-GA algorithm by combining the desirable characteristics of FA and GA. The emergency logistics model of this paper includes location decisions and allocation decisions. Considering the characteristics of FA and GA algorithms, we plan to use FA to solve location decisions and use GA to solve allocation decisions. Before presenting the detailed implementation of the proposed hybrid algorithm, we give some schemes for improving the algorithm efficiency.

### 3.4. Schemes for Improving the IFA-GA Algorithm

Most of the metaheuristic algorithms would suffer from two problems: metaheuristic algorithms usually have an earlier convergence, and the initial solution and the diversity of the solution space often affect their search quality. To overcome these two shortcomings, we enhance the proposed IF-GA algorithm through three schemes in this section.

#### 3.4.1. Scheme 1: Population Initialization

The initial population has a significant effect on the convergence speed and the quality of the final solutions. In most metaheuristic algorithms, a population is generated by random initialization. In this paper, we initialize the population by a myopic strategy.

Suppose RTCs can be located at any point of two-dimensional space with the cardinality constraint that the total number of RTCs is no more than *I*. First, the LDPs are clustered into *I* groups by considering the weight of demand. The locations of RTCs are selected at the center of gravity in each group. Then, we get a solution $\overset{⟶}{z}=\left[z_{1},z_{2},\ldots ,z_{I}\right]$. The population of location decisions is generated by random initialization around $\overset{⟶}{z}$. Second, for each location decision, allocating the resources according to the proportion of demand, we can obtain an even solution $\overset{⟶}{x}=\left[x_{o1},x_{o2},\ldots ,x_{oI}\right]$, $\overset{⟶}{y_{1}}=\left(y_{ij1}\right)$, and $\overset{⟶}{y_{2}}=\left(y_{ij2}\right)$. Select two elements of $\overset{⟶}{x}$ randomly. The first element subtracts a random number which is added to the second element. The random number is not bigger than the first element. The corresponding rows of $\overset{⟶}{y_{2}}$ should be changed accordingly. For $\overset{⟶}{y_{1}}$, we introduce a random matrix $\overset{⟶}{w}=\left(w_{ij}\right)$, each row of $\overset{⟶}{w}$ only has two nonzero elements in random columns with a random value $\tilde{w}$ and $-\tilde{w}$. Adding $\overset{⟶}{y_{1}}$ to $\overset{⟶}{w}$, we obtain a new $\overset{⟶}{y_{1}}$. Finally, the initial population is obtained by repeating the above process.

The article "A Novel Hybrid Algorithm for Multiobjective Location-Allocation Problem in Emergency Logistics" was retracted in 2023. Reasons: unreliable results or conclusions; concerns about the data; concerns about the results or conclusions; concerns about the peer review.

#### 3.4.2. Scheme 2: The Improved Search Strategy of FA

In this paper, FA is used to solve the facility location decision of RTCs. As is mentioned above, each decision variable *z*_*i*_ has a corresponding position. To be more realistic, we do not constrain the positions and only consider a cardinality constraint of RTCs. Therefore, we use coordinate variable *X*_*i*_=(*p*_*i*_^*x*^, *p*_*i*_^*y*^) to replace *z*_*i*_ for simplification and define *X*=[*X*_1_, *X*_2_,…, *X*_*I*_]. The objective function determines the fitness of firefly *X*. The direction and brightness of fireflies depend on the Euclidean distance between them and their fitness.

A dimmer firefly (worse solution) will be attracted by a brighter one (better solution) in FA. This mechanism is beneficial to the convergence of the algorithm. Thus, FA can find the optimal solution quickly. However, FA may fall into premature convergence if it encounters local extrema because the incomplete exploration of nondominated fireflies is one of the main reasons to cause the local convergence of FA. To overcome this weakness, we introduce a new update function for nondominated fireflies, described as follows:

(26) $$\begin{array}{c} X_{n+1}=X_{n}+\alpha_{n}\left(\varepsilon_{n}-0.5\right)X_{M}, \end{array}$$

where *X*_*M*_=*X*_Max_ − *X*_*n*_ if *ε*_*n*_ > 0.5 and *X*_*M*_=*X*_*n*_ − *X*_Min_ if *ε*_*n*_ < 0.5. *X*_Max_ is the upper bound of search space, and *X*_Min_ is the lower bound. Furthermore, for dominated fireflies, we consider the attraction of the best solution, and the iterative equation is modified as follows:

(27) $$\begin{array}{c} X_{n+1}=X_{n}+\beta_{0}e^{-\gamma r^{2}}\left({\tilde{X}}_{n}-X_{n}\right)+\beta_{0}e^{-\gamma r_{\text{opt}}^{2}}\left({\tilde{X}}_{\text{opt}}-X_{n}\right)+\alpha_{n}\varepsilon_{n}, \end{array}$$

where ${\tilde{X}}_{\text{opt}}$ is the brightest firefly in population and *r*_opt_ is the distance between ${\tilde{X}}_{n}$ and ${\tilde{X}}_{\text{opt}}$.

The article "A Novel Hybrid Algorithm for Multiobjective Location-Allocation Problem in Emergency Logistics" was retracted in 2023. Reasons: unreliable results or conclusions; concerns about the data; concerns about the results or conclusions; concerns about the peer review.

#### 3.4.3. Scheme 3: The Update Mechanism of Population

A good algorithm should have an excellent performance in exploring the solution space and have a good ability in convergence. In this paper, the IFA is nested into GA for solving the location problem. GA already has an elimination mechanism that replaces poor solutions to maintain the size of the population. However, the number of eliminated solutions is usually fixed in the original GA. Reference [25] proposed an adaptive mechanism to replace poor solutions dynamically. The number of eliminated solutions decreases in the iterative process. Therefore, the algorithm first tends to explore the solution space better and then moves to the local search. With the same purpose, we introduce the mutated number of GA as follows:

(28) $$\begin{array}{c} q=\left\lceil \text{rand}\left(\left.0,1\right)\right){}^{*}\text{PS}{}^{*}\left(1-\frac{t}{G_{\text{MAX}}}\right)\right\rceil , \end{array}$$

where ⌈⌉ is the ceiling operator, PS is the population size, *t* is the current number of iterations, and *G*_MAX_ is the maximum number of iterations.

The procedure of IF-GA is described in Algorithm 1 in detail.

## 4. Numerical Studies

In order to illustrate the proposed model and validate the performance of IFA-GA, a small-scale instance with one SNS, 10 RTCs, and 40 LDPs is first used. Although the number of nodes in emergency logistics is not considerable, the proposed model has 820 (2 *∗* 10*∗* 40 + 10+10) decision variables. It is an extremely complex optimization problem. The results with different objective functions are presented to show the decision differences related to deprivation costs. Furthermore, a comparison is made between IFA-GA, FA, GA, and particle swarm optimization (PSO) based on the same population initialization. The adjustment method for the infeasible solutions in Algorithm 1 is also used in each algorithm to satisfy the constraints *t*. Finally, instances extracted from large-scale disasters are used to demonstrate the effectiveness of the designed IFA-GA algorithm furtherly. All experiments are implemented using MATLAB 2019 on a ThinkPad T460s laptop with Intel i5-6200u CPU, 2.3 GHz frequency, and 12 GB memory.

The article "A Novel Hybrid Algorithm for Multiobjective Location-Allocation Problem in Emergency Logistics" was retracted in 2023. Reasons: unreliable results or conclusions; concerns about the data; concerns about the results or conclusions; concerns about the peer review.

### 4.1. Parameter Setting

In this experiment, we initialize the affected areas in a 100*∗*100 two-dimensional space randomly. The demand of each affected area is sampled uniformly in [50,150]. We assume that the RTCs can be located at any point of the space; then, the distance between a selected RTC and the other node is easily calculated by the Euclidean distance equation. The cost parameters and other variables in the proposed model are shown in Table 1.

It is essential to select suitable parameters for metaheuristic algorithms. Additionally, to evaluate the performance of the proposed IFA-GA, we compare it with the standard FA, GA, and PSO. The parameter settings of these algorithms are displayed in Table 2.

### 4.2. Computational Results regarding Deprivation Costs

As discussed above, the deprivation cost is an essential factor for the relief decision. To visually illustrate its impact on decision-making, we analyze the location results of RTCs which are shown in Figure 1. Because each RTC is linked to SNS, which is located at point (0,0) in our setting, we ignore the paths between SNS and RTCs for simplification. Figure 1 has six pictures. The first three pictures (a), (b), and (c) present the RTCs' locations with a single objective. The subsequent pictures present the RTCs' locations with two and three objectives. Obj1 refers to the deprivation cost objective. Obj2 refers to the unsatisfied demand loss. Obj3 refers to the operation cost. By comparing Figures 1(a) and 1(c), we can find that the locations of RTCs are closer to the affected areas in (a) than in (b). It is realistic because closer to demand will shorten the delivery time. In Figure 1(b), the locations are strange at first glance. It should be noted that objective 2 does not have any path-related cost, so the locations move randomly in the algorithm and have no practical meaning. Figures 1(d) and 1(e) confirm the random location results in (b), which have the same results as Figures 1(a) and 1(c), respectively.  Figure 1(f) shows the tradeoff location results by objective 1 and objective 3. Figure 1 illustrates that the deprivation cost impacts RTCs' locations, which makes RTCs closer to LDPs.

### 4.3. Computational Results of Different Algorithms

In this section, we further present several cases to illustrate the effectiveness of the proposed algorithm. For the small-scale case, the iteration results of IFA-GA, FA, GA, and PSD are shown in Figure 2. From Figure 2, we can see that the proposed IFA-GA has the best performance in both convergence and objective value. FA and PSD are almost unchanged because the flow balance constraints in the optimization model make the most newly generated solutions infeasible. GA has a certain convergence, but the objective values are much bigger than those of FA. It should be noted that FA, GA, and PSD are implemented with the same population initialization as IFA-GA. If the population are initialized randomly, the results of FA, GA, and PSD will be much worse.

The article "A Novel Hybrid Algorithm for Multiobjective Location-Allocation Problem in Emergency Logistics" was retracted in 2023. Reasons: unreliable results or conclusions; concerns about the data; concerns about the results or conclusions; concerns about the peer review.

To compare the results detailedly, we carry out each algorithm 30 times. More detailed results are given in Table 3. From Table 3, we can find that the proposed IFA-GA has better performance than the other algorithms. The mean, max, and min values of the objective obtained by IFA-GA are less than in the other algorithms. The standard deviation of objective values in IFA-GA is much lower than in other algorithms. Furthermore, the run time of IFA-GA is also less than other algorithms. The results of Table 3 indicate that the IFA-GA has better stability and efficiency in solving our proposed model.

Additionally, we conduct experiments with different problem sizes. Four large-scale instances are experimented for further comparison. The results are shown in Table 4.

From Table 4, we can find that the proposed IFA-GA obtains solutions with the best performance than the other algorithms in each instance. In both four cases, IFA-GA obtains the minimum objective value and the lowest deviation. Furthermore, IFA-GA also has the shortest run time. These gaps are to increase along with the problem size increases. FA has the worst performance in run time and stability. GA outdoes FA in each case, with almost the same objective values as PSD but a much lower run time. Additionally, the increase in LDPs brings more objective costs, but the increase in RTCs takes lower objective costs. The result can be obtained by comparing the case *I*=20, *J*=100 with the case  *I*=50, *J*=100. The reason is that the increase in RTCs can reduce the deprivation costs effectively, which enlightens us that more RTCs are recommended to be established when faced with large-scale disasters.

Based on the simulation results, we can derive some practical implications. First, RTCs should be located closer to rescue demand to decrease the human suffering caused by deprivation. Second, in a large-scale disaster scenario, more RTCs should be established to provide fast relief. In the theoretical aspect, we validated the efficiency of the proposed hybrid algorithm, which has an excellent performance in convergence and computation time.

## 5. Conclusions

Different disasters have affected most areas of the world and caused serious casualties and property losses in recent years. An effective emergency logistics occupies a pivotal position to relieve human suffering and mitigate losses after disasters. This paper proposes a multiobjective optimization model for relief distribution. The relief supplies are transferred in a three-level logistics network which includes an SNS, some RTCs, and LDPs. The location decision of RTCs and resource allocation decision from SNS to RTCs and from RTCs to LDPs should be made in postdisasters. We present three objectives, deprivation costs, unsatisfied demand costs, and logistics cost, in this location-allocation optimization model, in which several cardinality and flow balance constraints are considered simultaneously. Realizing the complexity of the problem, we design a novel IFA-GA algorithm by combining classical FA and GA. Three schemes are proposed to improve the effectiveness of the IFA-GA algorithm. The results from numerical studies provide several insights on the theory and practice of relief distribution, which also illustrate the validity of the proposed solution algorithm.

The article "A Novel Hybrid Algorithm for Multiobjective Location-Allocation Problem in Emergency Logistics" was retracted in 2023. Reasons: unreliable results or conclusions; concerns about the data; concerns about the results or conclusions; concerns about the peer review.

This study is not exhaustive. We only present a simplified model and ignore some factors which will make the model more complex. For example, the uncertainty factors, such as delivery time and quantity, are not considered in the proposed model. Multiple transport and multiple periods are also not investigated in our model. Therefore, we may extend the proposed model to an uncertain situation by using robust optimization theory or distributionally robust theory for future work. Furthermore, more hybrid algorithms that combine exact and metaheuristic approaches should be exploited to solve the proposed optimization model effectively in the future.

## Figures and Tables

**Figure 1:** The comparison of location decision with the different objective function. (a) Obj1. (b) Obj2. (c) Obj3. (d) Obj1 + Obj2. (e) Obj2 + Obj3. (f) Obj1 + Obj2 + Obj3.

**Figure 2:** The comparison of objective values obtained by different algorithms.

**Algorithm 1:** IFA-GA.

**Table 1:** The values of parameters.

Notation	Value
*O*	1
*I*	10
*J*	40
*v*	20
*a*	2
*b*	100
*C*_*OI*_	0.08
*C*_*IJ*_	0.1
*C*_*i*_	1000
*CV*_*i*_	0.5
*Q*_*o*_	2000
*Q*_*i*_	100

**Table 2:** The parameter settings of algorithms.

Algorithm	Parameter	Value
IFA-GA	Population size	200
	Number of iterations	300
	Maximum attractiveness *β*_0_	0.1
	Absorption parameter *γ*	0.001
	Crossover probability	0.5
	Mutation probability	0.2

FA	Population size	200
	Number of iterations	300
	Maximum attractiveness *β*_0_	0.1
	Absorption parameter *γ*	0.001

GA	Population size	200
	Number of iterations	300
	Crossover probability	0.5
	Mutation probability	0.2

PSO	Population size	200
	Number of iterations	300
	Social acceleration coefficient	2
	Personal acceleration coefficient	2

The article "A Novel Hybrid Algorithm for Multiobjective Location-Allocation Problem in Emergency Logistics" was retracted in 2023. Reasons: unreliable results or conclusions; concerns about the data; concerns about the results or conclusions; concerns about the peer review.

**Table 3:** Numerical results on the small-scale instance.

Algorithm	Mean	Max	Min	STD	Time
IFA-GA	11641	11780	11529	91	51
FA	26246	26972	25586	555	409
GA	23685	23480	23994	191	123
PSO	22468	22242	22838	225	413

**Table 4:** Numerical results under different problem sizes.

Problem size		IFA-GA	FA	GA	PSO
*I*=20 *J*=50	Mean	17935	31047	28452	27439
	Max	18240	32567	29497	27883
	Min	17620	30021	27111	27037
	STD	264	1083	889	363
	Time	73	1193	159	607

*I*=20 *J*=100	Mean	124675	209152	190568	190039
	Max	125200	211813	192749	191352
	Min	124310	204755	187603	188398
	STD	352	2703	1874	1178
	Time	91	1487	198	756

*I*=50 *J*=100	Mean	78051	130882	119106	118934
	Max	79890	135157	122993	122101
	Min	75788	127140	115843	115521
	STD	1467	3048	2574	2338
	Time	139	2071	315	1087

*I*=50 *J*=150	Mean	179260	302016	290526	278969
	Max	181800	310912	296233	283487
	Min	177400	291990	287331	274882
	STD	1600	6886	4250	3687
	Time	215	3470	498	1876

## Data Availability

The data were included in the manuscript.
